# A Retrospective Study of Recurrent Bacterial Meningitis in Children: Etiology, Clinical Course, and Treatment

**DOI:** 10.1155/2022/3681871

**Published:** 2022-03-10

**Authors:** Xin Li, Hua-Zhang Liu, Ling-yu Pang, Xin Wen, Su-Zhen Sun

**Affiliations:** ^1^Department of Neurology, Children's Hospital of Hebei, Shijiazhuang 050031, China; ^2^Department of Pediatrics, The First Affiliated Hospital of Shandong First Medical University & Shandong Provincial Qianfoshan, Jinan 250014, China; ^3^Department of Otolaryngology, Children's Hospital of Hebei, Shijiazhuang 050031, China

## Abstract

**Objectives:**

Recurrent bacterial meningitis (RBM) is a rare but life-threatening disease. This study aims to analyze the clinical features, potential causes, and therapeutic outcomes of RBM in children.

**Methods:**

This article retrospectively reviews the clinical characteristics, etiologies, and treatments in children with RBM hospitalized in Hebei children's hospital from 2012 to 2020.

**Results:**

A total of 10 children with RBM, five males and five females, were included in this study. The age of RBM in children spans from the neonatal stage to the childhood stage. The underlying illnesses were identified and classified as cerebrospinal fluid rhinorrhea (1 case), humoral immunodeficiency with Mondini dysplasia (1 case), common cavity deformity with cerebrospinal fluid ear leakage (1 case), Mondini malformations (2 cases), incomplete cochlear separation type I with a vestibular enlargement (2 cases), local inflammation of the sphenoid bone caused by cellulitis (1 case), congenital skull base defects (1 case), and congenital dermal sinus with intraspinal abscess (1 case). 6 patients chose targeted therapy for potential reasons.

**Conclusions:**

Congenital abnormalities or acquired injuries lead to intracranial communication with the outside world, which can quickly become a portal for bacterial invasion of the central nervous system, resulting in repeated infections.

## 1. Introduction

Recurrent bacterial meningitis (RBM) is defined as any reappearance of clinical and laboratory signs and symptoms of bacterial meningitis after adequate and successful treatment of a preceding meningitis [1, 2]. The causes of RBM in children are complex and diverse. Children's nervous systems undergo rapid structure and function development; therefore, the etiology often involves congenital structural abnormalities, adjacent organ infections, encephalopathy complications, immunodeficiency, etc. [3]. The treatment of RBM depends on the underlying cause and always involves antibiotics. The exact incidence of recurrent bacterial meningitis is not known. In 2019, a multicenter study of children with recurrent pneumococcal meningitis showed an incidence of 1.5% [4]. A recent study showed that RBM incidence in children in Beijing, China, was 2.3%, which is relatively uncommon [5]. This study analyzed the clinical manifestations, auxiliary examination, and therapeutic outcomes of 10 Chinese children with RBM admitted to Hebei Children's Hospital from 2012 to 2020.

## 2. Methods

From January 2012 through December 2020, 10 children with RBM were identified in Hebei Children's Hospital. The criteria for definite diagnosis of RBM [2, 6] include clinical presentations (fever, headache, vomiting, mental changes), positive cultures of cerebrospinal fluid (CSF) and/or blood, and other CSF laboratory findings (CSF leukocyte count >1000/mm^3^, predominantly polymorphonuclear cells; CSF glucose <50% of blood glucose; CSF protein of >50 mg/dl).

The second episode of meningitis is caused by a different pathogen than the first. If it were due to the same pathogen, the next episode would occur more than 3 weeks after completing therapy for the previous episode [1, 2, 7].

Patients excluded from this study were those who presented to the neurosurgery department due to trauma and not to the neurology department.

We collected the data from medical records to determine the age of the first onset episode of meningitis, the number of episodes, types of organism, clinical manifestations, investigations performed, the underlying causes of recurrence, treatment, and the total follow-up period. The institutional review board committee (IRB) of the Hebei Children's Hospital (123) has approved this study.

### 2.1. Statistical Analysis

Categorical variables were expressed as numbers and percentages. Continuous variables (normal distribution) were expressed as mean ± standard deviation (SD).

## 3. Results

In the study, from 2012 to 2020, we collected the data of 786 children with bacterial meningitis from the medical records of the Hebei children's hospital. We then enrolled 10 subjects identified with recurrent meningitis: five males and five females. The rate of RBM in children was 1.27% (10/786). The baseline characteristics of these 10 patients and their clinical manifestations are listed in Table 1.

The mean patient age was 50 months (range:1-108 months). The mean follow-up time was 20 months (range: 6-36 months), and the total number of meningitis episodes was 32, ranging from 2-5 episodes per patient.

All the patients had a fever (body temperature 38-40°C) and an altered mental status, but no convulsions. The onset time ranged from 4 hours to 7 days. Headaches and projectile vomiting always occurred in older children, whereas babies had irritability and bregma bulging. Meningeal irritation was positive in eight cases (72.7%), all of which were children over 3 years of age.

Of the 32 meningitis episodes, only 26 episodes had detailed results. Peripheral blood studies revealed a C-reactive protein (CRP) ranging from 1.1-379 mg/L, a (10.5-34.1) ×109/L white-cell count, and neutrophils (55%-98%). Serum immunoglobulins and total lymphocyte immunity analysis were performed in 6 patients. 1 case had abnormalities with IgM, IgA, and IgG at 0.01 g/L 0.01 g/L, and 0.02 g/L, respectively, and were considered as X-linked agammaglobulinemia.

Blood culture was tested for all patients, with 6 patients (54.5%) positive for bacteria. Of which *S. pneumonia* was found in 5 cases and *Haemophilus influenza* (*H. influenzae*) in 1 case. Pathogens grown from blood cultures were identical to those from CSF cultures. All patients had at least one positive CSF culture, but only one organism was detected in the same patient. Of the 10 cases, the bacteria identified in the CSF cultures were *S. pneumonia* in 8 cases (80%), *H. influenza* in 1 case (10%), and *staphylococcus aureus* (*S. aureus*) in 1 case (10%). The primary causative agent identified from the CSF cultures was *S. pneumoniae*. The CSF glucose levels ranged from 0.01 to 2.87 mmol/l, total protein from 0.23–3.4 g/L, lactate from 5.06-18.8 mmol/L, and a WBC count of (0.55 –11.41) ×109/L.

Computerized tomography (CT) scans of the temporal bone were available for 9 patients, 7 of whom showed abnormal images, including 6 inner ear deformity cases and 1 local bone destruction case. The types of inner ear malformations in 6 patients were: common cavity deformity with cerebrospinal fluid ear leakage (1 case), Mondini malformations (3 cases), incomplete cochlear separation type I with a vestibular enlargement (2 cases). All children were examined by cranial magnetic resonance imaging (MRI), of which 4 had abnormal brain parenchymal signals, and one case showed discontinuous skull base lamina bone cortex and local encephaloceles (Figure 1). 8 cases underwent whole spinal cord MRI, and 1 case had sacrococcygeal hairy sinus with intraspinal abscess (Figure 2).

All the patients were healthy before the first episode of meningitis. Of the 10 patients, 2 patients had congenital deaf-mutism. 1 patient had eye cellulitis before suffering from bacterial meningitis and inflammatory lesions in the nasal bone even after the first infection was cured (Figure 3), and 1 patient had a history of falling from a 2-story height.

All patients were treated with a combination of ceftriaxone and vancomycin. Antibiotics were adjusted based on the cerebrospinal fluid culture results. The case considered as X-linked agammaglobulinemia was treated with immunoglobulin intravenously every 21 days. None of the patients received prophylactic antibiotic treatment. Six of ten patients with anatomical defects underwent corrective neurosurgical operations.

The total follow-up period ranged from 6 months to 3 years. Death due to meningitis was not reported. Neurological consequences related to meningitis included global developmental delay in 2 (20%) patients. 4 patients (40%) who had sensorineural hearing loss were mainly related to their original disease.

## 4. Discussion

RBM in children is a rare disease since the subarachnoid space is adjacent to the sinuses, nasopharynx, middle ear cavity, skull, and skin. Congenital abnormalities or acquired injuries allow the subarachnoid space to communicate with these structures and can easily become a gateway for bacterial invasion of the central nervous system, leading to repeated infections [2, 8, 9]. Tebruegge et al. concluded that common causes were anatomical problems (59%), immunodeficiency (36%), and para-meningeal infections (5%) [1].

In this study, we reported on 10 children with RBM. In our series, the causes of RBM were all related to anatomical problems. Congenital abnormalities (80%) included congenital inner ear malformation (60%), skull base cortical bone discontinuities (10%) and dermal sinuses (10%). Acquired injuries (20%) include trauma (10%) and infection (10%). Only 1 child had congenital inner ear malformation combined with X-linked agammaglobulinemia.

Patients with inner ear malformations have an increased risk of developing bacterial meningitis [10–12]. Abnormal inner ear development leads to a channel between the tympanic cavity and the subarachnoid space [1, 10]. CSF flows out through this channel, forming a CSF otorrhea through which pathogens enter the intracalvarium and cause purulent meningitis [13–15]. The organisms reported in meningitis due to inner ear malformation and CSF leaks include *S. pneumonia*, *H. influenza*, and *S. aureus* [1, 16–18]. In our study, 9 children underwent temporal bone CT; 7 cases were abnormal with a more than 50% positive rate. Among them, there were 6 cases of inner ear malformations. *S. pneumoniae* was the most common meningitis pathogen, accounting for 80% of inner ear malformations cases, followed by *H. Influenza* (20%). It is worth noting that two children with inner ear malformations had congenital deaf-mutism. Therefore, for congenital deaf-mute children with first purulent meningitis, temporal bone CT or inner ear MRI must be performed to determine the presence of otorrhea [10, 19]. Considering that inner ear malformation is an autosomal dominant genetic disease, special attention should be paid to hearing screening and temporal bone CT if children with first-onset purulent meningitis have a family history of deafness [20]. Surgical correction of the inner ear malformation or defect is necessary to prevent recurrent pyogenic meningitis [21, 22]. Unfortunately, surgical intervention was not performed in all patients. 2 patients chose conservative treatment due to the charge and the risk of the operation.

Immune factors are also one of the reasons that lead to recurrent brain transformation that cannot be ignored. Children with congenital immunodeficiency syndromes tend to present with recurrent meningitis in late childhood and early adulthood [1, 23]. Complement deficiency has been reported to increase the susceptibility to meningococcal disease and repeated infections [24, 25]. Some researchers recommend that all children with RBM be screened for primary immunoglobulin or complement deficiencies [26]. Among the cases we counted, one child had inner ear malformations and 2 episodes of bacterial meningitis in six months with *H. influenza* present in the CSF was culture. Immunoglobulin tests showed a complete reduction of IgG, IgM, and IgA and 0% of CD19^+^ cells, which was considered as X-linked agammaglobulinemia [27]. The child received regular monthly intravenous immunoglobulin and was followed up for 1 year without meningitis recurrence. When clinicians encounter prolonged and repeated encephalitis, they need to be alert to whether they are associated with immune system-related diseases.

In our series, other congenital causes of RBM include congenital dermal sinuses and congenital encephaloceles of the anterior skull base. A dermal sinus is an abnormality that appears above the dorsal midline at birth. An abnormal epithelialized connection extends from the skin towards the spine and is most commonly seen in the lumbosacral and occipital regions [28, 29]. There are often abnormal hair, pigmentation or capillary tumor-like changes around the sinuses, which can be found with the clinician's careful examination [30]. Infections can lead to periventricular abscess and intraspinal infection, causing RBM [22]. *S. aureus* is a common pathogen followed by *Escherichia coli* and anaerobic bacteria [31–33]. One case in our study had onset in infancy. The sinus was located in the lumbosacral region, so we could only see a little bit of hair without local redness or swelling. Spinal MRI suggested lumbosacral sinus, but the subarachnoid space signal was uneven. Sinusotomy showed the sinus tract was not connected to the spinal cord, but fever recurred after surgery. Reexamination of the child's cerebrospinal fluid revealed an abnormality with the spinal cord, and MRI revealed a spinal canal abscess. After resection of the abscess, no recurrence was observed for 2 years. The pathogen was confirmed as *S. aureus*. Therefore, attention must be paid to the physical examination of the first-episode purulent meningitis in infancy, especially in the neonatal period [4]. MRI of the whole spinal cord is also recommended to screen for hidden sinus and be alert for intraspinal abscess [31].

Congenital encephaloceles of the anterior skull base is a relatively rare abnormality in which a sac-like protrusion of intracranial contents herniates through a bony defect in the skull [34, 35]. Intracranial structures are protected by bone and dura mater, which is the most crucial barrier that reacts strongly in the face of an infection. Structural defects in these barriers facilitate the spread of infection to the subdural areas [36]. Since basal encephaloceles have less apparent external manifestations, their presentation may be more insidious, varying from nasal airway obstruction to frank meningitis of a wide age range [37]. One study showed that the vast majority of meningitis episodes in basal encephaloceles were caused by *S. pneumonia* (83%), followed by *S.aureus* (11%) and *N. meningitides* (6%) [1]. The case we reported was a 4-year-old boy who developed two episodes of bacterial meningitis within 5 months, with primary manifestations such as fever, headache, and vomiting. *S. pneumonia* was present in both of the cerebrospinal fluid cultures. Sinus CT showed discontinuity of the left skull base lamina bone cortex and local encephaloceles. After surgical repair of the lamina at the base of the skull, no recurrence of encephalitis occurred at 18 months follow-up.

Acquired structural abnormalities are more common in CSF rhinorrhea, otorrhea, or inflammatory tissue package caused by trauma and infection of adjacent tissues, such as cellulitis and otitis media. The underlying cause is a trans-dural communication between the meningeal space and paranasal sinuses or skin [38]. Bacterial penetration of the subarachnoid space may occur directly through a breach in the skull and adjacent soft tissues, which is the cause of meningitis [39]. Patients with head injury have the highest risk of acquiring recurrent bacterial meningitis [38]. Delayed recognition of the signs and symptoms of orbital cellulitis can lead to severe complications such as meningitis, cerebral abscess, and blindness [40]. It is known that the interval between trauma/infection and the first episode of meningitis varies from a few hours to many years [1, 2, 41, 42]. In our study, 1 child with head trauma developed intermittent nasal flow “clear water” within 1 year and four recurrences of bacterial meningitis within 1 year. The symptoms quickly relieved each time, always in 1-2 weeks. Cranial MRI revealed bilateral frontal lobe softening with glial hyperplasia, cerebrospinal fluid, and nasal fluid contrast showed approximately the same glucose, chloride, and protein levels, indicating cerebrospinal fluid rhinorrhea. The other patient in the study had first bacterial meningitis secondary to left eye cellulitis, and the sphenoid bone remained with the inflammatory lesions after the first infection was cured. The lesions resulted in recurrent bacterial meningitis in the patient, which occurred 4 times within 3 years. After removing the lesion, the encephalitis did not recur during the 2 years' follow-up. The other patient had 4 episodes of bacterial meningitis within 2 years. Head MRI revealed malformations of the inner ear and temporal bone, which is suggestive of cerebrospinal fluid otorrhea. After the cerebrospinal fluid otorrhea repair, the encephalitis did not recur in 2 years of follow-up. There were 5 cases of otitis media and 4 cases of sinusitis in all cases. We believe that inflammation of adjacent tissues may cause bacterial meningitis, but otitis media and sinusitis cannot be blindly determined as the source of bacterial meningitis infection. Therefore, it is necessary to clarify whether the adjacent tissues were connected to the brain parenchyma, and the sinus CT and temporal bone CT can help judge this [2, 22, 43].

## 5. Conclusion

Although RBM in children is a rare disease, it may cause severe neurological dysfunction. Infantile or school-age children with first-episode meningitis need to exclude congenital structural abnormalities and deserve the attention of clinicians. Post-traumatic meningitis in the first episode must consider whether or not the child has cerebrospinal fluid leakage. Detailed medical history, careful physical examination, and comprehensive examination are the golden clues for the early diagnosis of RBM in children. Once an anatomical defect is identified, surgery is recommended for patients with RBM.

## Figures and Tables

**Figure 1:** CT of the left skull base lamina bone cortex revealing discontinuous local encephaloceles.

**Figure 2:** The spinal cord MRI revealing an abscess in the spinal canal.

**Figure 3:** Brain MRI revealing inflammatory lesions in sphenoid bone after the first infection.

**Table 1:** Features of the Patients with Recurrent Bacterial Meningitis.

No.	Sex	Age at first episode (months)	No of episodes	Pathogen	Auditory evoked potential/auditory test	Etiology	Surgical treatment	Outcome
1	M	34 months	3	S. pneumoniae	Normal	Mondini dysplasia with vestibular enlargement	Yes	3 years
2	F	60 months	2	S. pneumoniae	Bilateral severe sensorineural hearing loss	Congenital deaf-mutism/bilateral inner ear malformations	No	1 year
3	F	72 months	5	S. pneumoniae	Unilateral severe sensorineural Hearing loss	Cochlea incompletely delimited typeIwith vestibular enlargement and loss of posterior and external semicircular canal	Yes	2 years
4	F	30 months	2	H. Influenzae	Mild hearing loss in the right ear	Mondini dysplasia, humoral immunodeficiency disease	No	1 year
5	F	58 months	4	S. pneumoniae	Normal	Local inflammation of the sphenoid caused by cellulitis	Yes	6 months
6	M	47 months	2	S. pneumoniae	Normal	The discontinuous cortex of skull base ethmoid plate	Yes	18 months
7	M	1 month	3	S.aureus	Normal	Lumbosacral pilonidal sinus, intraspinal abscess	Yes	2 years
8	M	108 months	4	S. pneumoniae	Normal	Cerebrospinal rhinorrhea	No	1 year
9	F	7.6 months	3	S. pneumoniae	Binaural hearing screening failed	Cochlea incompletely separated I with vestibular enlargement	No	10 months
10	M	68 months	4	S. pneumoniae	Unilateral severe sensorineural hearing loss	Common lumen deformity of the left inner ear and cerebrospinal leak	Yes	3 years

## Data Availability

The data used to support the findings of this study are available from the corresponding author upon request.
